This article has been retracted.

# Automatic COVID-19 Lung Infection Segmentation through Modified Unet Model

**DOI:** 10.1155/2022/6566982

**Published:** 2022-04-11

**Authors:** Sania Shamim, Mazhar Javed Awan, Azlan Mohd Zain, Usman Naseem, Mazin Abed Mohammed, Begonya Garcia-Zapirain

**Affiliations:** ^1^Department of Software Engineering, University of Management and Technology, Lahore, Pakistan; ^2^School of Computing, UTM Big Data Centre, Universiti Teknologi Malaysia, Skudai 81310, Johor, Malaysia; ^3^School of Computer Science, The University of Sydney, Sydney, Australia; ^4^College of Computer Science and Information Technology, University of Anbar, 11, Ramadi 31001, Iraq; ^5^eVIDA Laboratory, University of Deusto, Avda/Universidades 24, 48007, Bilbao, Spain

## Abstract

The coronavirus (COVID-19) pandemic has had a terrible impact on human lives globally, with far-reaching consequences for the health and well-being of many people around the world. Statistically, 305.9 million people worldwide tested positive for COVID-19, and 5.48 million people died due to COVID-19 up to 10 January 2022. CT scans can be used as an alternative to time-consuming RT-PCR testing for COVID-19. This research work proposes a segmentation approach to identifying ground glass opacity or ROI in CT images developed by coronavirus, with a modified structure of the Unet model having been used to classify the region of interest at the pixel level. The problem with segmentation is that the GGO often appears indistinguishable from a healthy lung in the initial stages of COVID-19, and so, to cope with this, the increased set of weights in contracting and expanding the Unet path and an improved convolutional module is added in order to establish the connection between the encoder and decoder pipeline. This has a major capacity to segment the GGO in the case of COVID-19, with the proposed model being referred to as “convUnet.” The experiment was performed on the Medseg1 dataset, and the addition of a set of weights at each layer of the model and modification in the connected module in Unet led to an improvement in overall segmentation results. The quantitative results obtained using accuracy, recall, precision, dice-coefficient, F1score, and IOU were 93.29%, 93.01%, 93.67%, 92.46%, 93.34%, 86.96%, respectively, which is better than that obtained using Unet and other state-of-the-art models. Therefore, this segmentation approach proved to be more accurate, fast, and reliable in helping doctors to diagnose COVID-19 quickly and efficiently.

## 1. Introduction

Since December 31, 2019, COVID-19 has been identified as a new coronavirus outbreak from Wuhan, a province in China. Infected cases were reported in both the international community and other Chinese cities within a few days. Because of the virus's speed and breadth of transmission, the World Health Organization (WHO) declared the severe acute respiratory syndrome coronavirus commonly known as COVID-19 outbreak a pandemic [1]. There were 125,000 cases reported to WHO from 115 countries and territories, while the number of cases reported outside China also nearly doubled within a couple of weeks, and the number of nations affected nearly tripled [2]. Statistically, 305,914,601 people worldwide tested positive for COVID-19 and 5,486,304 people died as a result up to 10 January 2022 [3, 4].

The most common COVID-19 symptoms include respiratory ailment, cough, flu, and fever, while for its part, computer tomography (CT) is a far better form of technology in terms of reliability, speed, and usefulness. As the virus broke out rapidly, assessment of COVID-19 needed to be automatic in the case of this particular pandemic [5]. Assessment and classification of COVID-19 are quicker using CT scans, insofar as its early detection is possible using CT images, although classification takes a lot of valuable time as this is done manually by expert radiologists. RT-PCR test results for COVID-19 take more than one day for the virus to be detected in the human body [6, 7]. Ground glass opacity (GGO) in CT images is considered to be a sign of COVID-19, and GGO in CT images takes on a fuzzy appearance, with opaque cerebral lesions being either uni-partite, bilateral, cortical, or distributed invasive lesions. The immediate diagnosis of COVID-19 was initially pivotal in controlling the spread of disease [8]. Manual assessment and analysis of CT scans by expert radiologists are time-consuming procedures while the severity and spreading rate demand automatic segmentation and detection in a fast pace environment [9].

In this study, we proposed a deep learning improved model based on UNet [10] that segments the ground glass opacification areas in a COVID-19 CT image dataset that is available to the public. Some difficulties occur in the segmentation of CT scans due to varieties in surface, location, and area of tainted regions. In the case of segmentation models, very small lesions and interconnected components that appear indistinguishable in CT images effectively generate a greater likelihood of false negatives. The ground glass limitation, which results in a small difference between the region of interest and background and fuzzy appearance, leads to difficulty in distinguishing the region of interest from a normal background when the division is being measured, and these factors influence segmentation performance. Our work has two objectives. First, we ascertain whether a more weighted module can be used inside a U-Net to enhance CT images lesion segmentation for limited labeled data, which is common in COVID-19 due to a lot of time-consuming manual masking of CT images. Second, we combine our new adaption of this module and increase the number of convolving layers in standard Unet architecture. The following are the main contributions made by the study.

1. This research addresses the problem of being unable to distinguish ROI from a normal background in deep learning segmentation and uses convolution layers and an E-D connected module in a simple and easy way.
2. The increase in convolution layers extracts the features at a fine level and boosts the propagation of features. The E-D module enlarges the receptive field, and the gradient disappearance (indistinguishable) problem is recouped through the E-D module.
3. The proposed Unet-like model improves the receptive field of the predicted region of interest, leading to more information being gained and the edge recognition ability of the model being magnified.
4. The quantitative results of the proposed model compared to the basic Unet approach and other state-of-the-art models makes its performance the best one.

The rest of the paper is organized as follows: Section 2 describes related work on segmentation techniques and particular segmentation techniques for COVID-19 CT scans.  Section 3 explains the method proposed and implemented. In Section 4, our model performance with state-of-the-art is discussed and Section 5 provides the conclusion drawn from our article.

## 2. Related Work

Deep Learning has a great capability to learn and provide solutions to state-of-the-art inventions and problems in different diseases efficiently in this new era. The segmentation of COVID-19 CT scans using deep learning approaches has a broad scope in terms of research.

### 2.1. Image Segmentation

Deep learning segmentation models have been matured in recent years, resulting in the development of numerous automatic systems essentially based on deep learning approaches. Semantic segmentation algorithms have also been advanced and are quick, and these algorithms are automated using medical and natural image applications. In recent years, segmentation performance of medical images has been improved from the fully convolutional network (FCN) technique to an improved convolving method version, known as dilated convolution [11]. The extensive changes in encoder-decoder pipeline architecture for image classification and segmentation has provided good results as follows: SegNet [12], ResNet [13], NnUnet [14], A2-Net [15], ShelfNet [11], and discriminative learning [16].

### 2.2. Segmentation Approaches for COVID-19 CT Scans

The TV-Unet model is a modified Unet model that uses regularization terms in its network and has detected and segmented pathological regions. The Basic Unet model was improved by tuning the hyperparameters and was subject to a comparative analysis of different parameters in a research study [17]. The study proposed a two-stage method to improve the Unet model by adding a residual block that was used to detect subareas and tiny lesions accurately. A two-stage cross-domain transfer learning method is proposed by applying the ResNet50. In the first stage, transfer learning is applied to the model level, while, in the second stage, data level transfer learning is applied. Each layer of Resnet50 is embedded with an enhanced channel attention component [18]. The study proposed a covTANet model to diagnose Covid-19, the severity of infection, and segmentation of infected lung lesions. A full convolution network and Unet approach were also used with few modifications to covTANet [19].

FractalCovNet architecture is proposed using fractal modules for segmentation, and this includes U-Net architecture with fractal blocks. This architecture followed the contracting and expansive path, and the contraction and expansion procedure was repeated to obtain the segmented output [20]. A Unet variation worthy of note known as CXAU-Net [21] convolution added up the value of receptive fields while the hybrid loss function improved model performance. The study [22] used progressive global perception and local polishing to build the network that could then segment infected areas in CT images. This approach applied to segmentation was in accordance with Unet architecture, with the study proposing a RTSU-Net that improved on structural relationships by introducing a nonlocal neural network module [23]. The study coped with a COVID-19 CT scans data shortage by focusing on increasing data size using the augmentation method along with the Unet model implementation for segmentation [24].

## 3. Proposed Methodology

### 3.1. Dataset Description

The annotated Medseg1 dataset from the dataset [25] contains 100 CT images of 40 COVID-19 patients. One mask class is ground glass opacity, the second is consolidation, the third is another pulmonary infection, and the fourth is the lung. Four labeled classes are used in this dataset: 1 = ground class opacity, 2 = consolidation and 3 = pulmonary effusions and 4 = lung. This dataset contains 474 images in total, including original CT scans, as shown in Figure 1. The color augmentation, noise augmentation and minoring, scaling, rotation, and elastic deformation were applied in the case of spatial augmentation.

In this dataset, there are 96 images with ground glass masks, 78 with consolidation mask images, 100 other lung and pulmonary mask images, and also 100 background mask images. According to research, ground glass opacity is the most relevant in the diagnosis of COVID-19, and so here, we focused our study on ground glass opacity mask images and other labeled classes that were not used in our work. Here in Figure 2, row 1 shows original CT scans, the second row shows ground glass opacity mask images, and the third row shows consolidation mask images.

### 3.2. Model Description

The proposed network design we describe in depth in this section is that of CNN model architecture. The customized CNN model features key distinctions between the previous work and the method suggested. Different techniques and models for semantic segmentation are based on convolution layers. Unet [12] architecture is comprised of an encoder and decoder symmetrically, with the encoder path involving two convolution layers at each downward step. A 3*∗*3 convolved operation was then conducted, and pooling operation of size 2*∗*2 and stride size of 2 was applied. Moreover, this process was repeated four times to collect spatial features of an image in an encoder. At first, the decoder followed the upsample operation to map the feature using the transposed convolution of size 2*∗*2, reducing the number of channels by half. Two convolution layers of size 3*∗*3 then followed the upsample operation. The feature map from the last block of the decoder undergoes a 1*∗*1 convolution operation that produces the segmentation map of the same size as the input image. Unet architecture uses the RELU activation function throughout its convolution layer, while the last convolving layer uses the Sigmoid function.  Figure 3 shows the architecture of the proposed convUnet method.

Our proposed model is based on conventional Unet [12] architecture with the following enhancements:

1. The addition of convolution layers at each block of encoder structure and the same number of convolution layers are applied at each block of the decoder pathway. Both contraction and expansion paths have more sets of weights than Unet.
2. The set of weights in the encoder and decoder connecting module is increased from 2 to 3. The conventional Unet has 2, while our improved model has 3 sets of weights.
3. The improved model used Batch normalization before each nonlinear function. The conventional Unet has no use for batch normalization in its network.

This research increased the convolution layers in each block of encoder and decoder architecture. To optimally handle the input image dimension 512*∗*512, we used a U-Net structure from [19], which was slightly altered by adding one more convolving layer in each block of encoderand decoder. In our proposed model, there were four blocks that made up the downsampling path, while a further four blocks comprised the upsampling path. Three times 2D convolution with a kernel size of 3*∗*3, three times batch normalization, and three times the Relu activation function is used for each block of the encoder and decoder pipeline, while a 2D convolution with kernel size 1*∗*1 is used in the last block. In order to halve the spatial dimension of the feature maps after each block, a max-pooling operation is applied for downsampling. To double the size of the spatial dimension of the concatenated feature maps, ConvTranspose2d is used in the decoder pathway. In the downsampling path, the number of feature channels is increased to 1-64-128-256-512, and in the up-sampling path, it is reduced again from channel number 512 to channel number 1.  Figure 4 shows the flow of input images through the encoder pipeline. Each block shows which operation and how many convolution layers are used.

Figure 5 demonstrates the flow more clearly. The input image is convolved along with the use of batch normalization and nonlinear function, which reduces the channel number. It is then followed by a max-pooling operation to obtain a pooled feature map. Downsampling reduces the size of the input, and this sequence of operations is repeated four times in the encoder path.

Through skip connection, the output of each block comprising convolution layers that are obtained before the pooling operation in the encoder is passed to the corresponding decoder block. Furthermore, it becomes concatenated with the output of the transpose convolution layer, and feature maps are transferred to the decoder convolution layers. Feature information lost in the symmetric encoder due to the pooling operation can be obtained through skip connection, which enables the proposed model to use fine-grained details learned in the encoder part in order to construct an image in the decoder part. To summarize, the purpose of these skip connections used in the proposed model is that they provide an unvarnished or nonfluctuated gradient flow from the first to the final layer. The research supplemented a module in the Unet architecture as an addition to the U-bottleneck, which allowed us to gather contextual information just from the useful global context information required both proficiently and systematically, with the module structure being shown in Figure 6.

The output from the last layer of the encoder with small dimensions is taken as input to the more weighted connected module. This forms the local representation of feature maps that are produced from the final block of our proposed convUnet encoder path. The integrated module is placed into the bottleneck because the input passing through the module will have decreased in both size and dimension, reducing the amount of time spent on training and space complexity on the feature maps. Our customized model improves the segmentation performance on the COVID-19 dataset by increasing the number of convolution layers and modifying the connected encoder and decoder module that we added to the model.

Figure 6 represents the encoder-decoder-connected module. The last pooled feature map is passed through the module which has convolving layers of 3*∗*3 filter size.

The last layer feature map in our proposed model was in accordance with the soft-max classifier that generates a number of feature channels equal to the number of semantic segmentation label classes. The last layer obtained the image size 512*∗*512 equal to the actual image size with 4 channels, while the architecture had 46,773,124 parameters and 46,755,460 trainable parameters in total. Every convolution layer comprises feature maps, C represents the convolution layer, the feature map is denoted by *M,* and the layer number is denoted by *n*. The feature map in the first layer *C*^1^ derives from convolving the input matrix by a kernel *k*^1^ along with the addition of bias term *B*^1^. In this case, *j* denotes the feature map number and *f*(*y*), a nonlinear function, is applied to the filtered output before passing it on to the convolution layer, where I denotes the input neuron. Convolution at layer one with its elements is expressed in the following equation:

(1) $$\begin{array}{c} C_{j}^{\left(1\right)}=f\left(B_{j}^{\left(1\right)}+K_{j}^{\left(1\right)}\times I\right)\text{ where}\;j=1,\ldots ,M^{\left(n\right)}. \end{array}$$

In the first convolution layer *C*^1^, Input *I* is convolved with a weight matrix to obtain a feature map. The *M*1 feature map is obtained through sliding over the different positions of the input matrix according to the set value of stride. Features are extracted in this way, and thus, the weight parameters are shared for all infection classes in the case of our dataset (ground-glass opacity, consolidation, pulmonary). Therefore, the layer acquires an equivariance property and becomes invariant to the image transformation.

It also results in a sparse weight that leads to small, fine feature detection. Further layers are added to extract fine features from starting layers. The feature map at different levels and at different layers can be expressed as follows:

(2) $$\begin{array}{c} C_{j}^{\left(n\right)}=f\left(B_{j}^{\left(n\right)}+\sum_{i=1}^{r\left(n-1\right)}K_{j}^{\left(n\right)}\times r_{i}^{\left(n-1\right)}\right)\text{where}\;j=1,\ldots ,M^{\left(n\right)}. \end{array}$$

Table 1 shows the difference between the conventional Unet and proposed convUnet models. In the whole network, Unet includes 16 convolution layers, while the proposed model is comprised of 24. The Unet consists of 2 sets of weights in its connected module, while the proposed one has 3. Lastly, Unet does not include batch normalization, while the proposed model did use it.

### 3.3. Loss Functions

The dice coefficient-based loss function was used per 100 epochs to express dice loss, the latter also being included in the evaluation matrix.

(3) $$\begin{array}{c} \mathrm{Dice}\;\mathrm{loss}=1-\mathrm{dice}\left(a,c\right)=1-2\times \frac{a\cap c}{a+c}. \end{array}$$

#### 3.3.1. Binary Cross Entropy

The last layer in our proposed model follows the Unet approach that generates a number of feature channels equal to the number of semantic segmentation label classes. Our dataset contains multilabel classes, and so we used the soft-max function with binary cross entropy for loss function. In the last layer, we obtained an image size of 512*∗*512 equal to the actual image size with 4 channels.

The binary cross entropy is used as follows:

(4) $$\begin{array}{c} \mathrm{BCE}=-\frac{1}{n}\overset{n}{\underset{i=1}{\sum }}\left[y_{i}\log\left(y_{i}^{\prime }\right)+\left(1-y_{i}\right)\log\left(1-y_{i}^{\prime }\right)\right]. \end{array}$$

For multilabel classes, the binary cross entropy, where *o* = 4, is as follows:

(5) $$\begin{array}{c} \mathrm{BCEM}=-\frac{1}{n}\overset{n}{\underset{i=1}{\sum }}\overset{o}{\underset{k=1}{\sum }}y_{\mathrm{ik}}\log\left(y_{\mathrm{ik}}^{\prime }\right). \end{array}$$

### 3.4. Implementation Details

The convUnet model proposed in this article was implemented in Google colab using python language, while convUnet training and testing were done using an Intel(R) Core (TM) i3-4030U CPU @ 1.90 GHz 1.90 GHz 64-bit operating system. To train the data, we selected the “adam” optimizer as an optimization technique. The test size for the data was set to 20%, and the input image size for training data was 512*∗*512 with a batch size of 1 per 100 epochs and a learning rate of 1*e* − 3.

## 4. Results

This section provides the results obtained and discussion on the results in detail, providing both quantitative and qualitative results obtained using the improved model and a quantitative comparison between the improved model with other models and with the baseline approach. We used the following performance measure metrics to measure the performance of the improved model.

### 4.1. Segmentation Evaluation Index

Accuracy (1) is the ratio between the sum of true prediction of both (positive and negative results) and the sum of all false and true predicted values.

(6) $$\begin{array}{c} \text{accuracy}=\frac{TP+TN}{TP+TN+FP+FN}. \end{array}$$

Sensitivity (2) is the ratio between correctly predicted segmentation and the sum of correctly predicted segmentation and false prediction as nonlesion. In medical studies, sensitivity is critical. The lower the sensitivity, the higher the occurrence of false-negative prediction. In the case COVID-19, if a person with it is predicted “negative,” this can be caused by the further spread of the virus. Thus, model sensitivity must be high in the case of the efficient model.

(7) $$\begin{array}{c} \text{Senstivity}=\frac{TP}{TP+FN}. \end{array}$$

Precision (3) is the ratio between correctly segmented prediction and total predicted segmentation.

(8) $$\begin{array}{c} \text{Precision}=\frac{TP}{TP+FP}. \end{array}$$

Specificity (4) is the ratio between true negative and the sum of true negative and false positive.

(9) $$\begin{array}{c} \text{Specificity}=\frac{TN}{TN+FP}. \end{array}$$

*F*1 score (5) is the ratio between the two times multiplication of precision and sensitivity multiplied result and the sum of precision and sensitivity.

(10) $$\begin{array}{c} F1\text{ score}=2\times \frac{\text{Precision}\times \text{Senstivity}}{\text{Precision}+\text{Senstivity}}. \end{array}$$

Dice coefficient is the ratio between two times multiplication of the intersected value of actual value and predicted value of the model and the sum of actual value and predicted value.

(11) $$\begin{array}{c} \text{Dice co}-\text{efficient}=2\times \frac{a\cap c}{a+c}. \end{array}$$

Jaccard index: Jaccard index, which is commonly known as intersection over union (IOU), measures the similarity between actual ground truth and predicted segmentation. It refers to the intersection area of GT and PS divided by the union of both GT and PS.

(12) $$\begin{array}{c} IOU\left(a,c\right)=\frac{\left(a\cap c\right)}{a\cup c}. \end{array}$$

Here, *a* and *c* show ground truth value and predicted value, respectively.

In Figure 7, the a and c columns represent the actual ground truth of ground glass opacity, while the c and d columns represent predicted segmentation by our model.

### 4.2. Qualitative Analysis

Figure 8 shows some of the findings acquired for ground glass opacity area segmentation by displaying the ground truth and the results provided. Our suggested approach produced good segmentation results without using complex models. In addition, when compared to ground truth, we obtained good segmentation compared to other models in our study. Figure 8 shows some instances of the findings acquired with a view to evaluating the performance of the proposed approach for segmentation of the lung infection area at ground glass opacity level. In Figure 8, the first column represents the original CT scan, the second represents the actual ground truth, and the third shows our segmentation results. We can see from the data that the suggested model identified the ground glass opacity well with certain mistakes that are considered insignificant. Furthermore, as shown in Figure 7, the segmentation results obtained from our model are close to the actual ground truth.

### 4.3. Quantitative Results

Table 2 shows the quantitative results of the proposed model and baseline approach Unet model. Our model obtained the best results in terms of dice coefficient, Jaccard index, recall, F1 score, and precision with scores of 93.29, 92.46, 86.96, 93.01, 93.34 and 93.67, respectively. For its part, the proposed convUnet model obtained an average result over 100 epochs of 76.47%, 83.27%, 82.52%, 83.43%, 82.75%, and 84.11% in the case of IoU, accuracy, dice coefficient, *f*1-score, recall, and precision, respectively.

Figure 9 shows the box plot of the proposed model results for accuracy, dice coefficient, intersection over union, precision, *F*1-score, and recall. Each color indicates different performance measure metrics. The boxes' upper and lower boundary represents the range of result scores, while a line in the same color inside the colored box refers to the average score, which falls between 0.8 and .09 in the case of all evaluation indexes mentioned. The results below the whiskers represent outliers, which are shown as colored dots.

Figure 10 represents the training and testing performance of the proposed model over 100 epochs. It can be noticed that in early epochs, the difference between training and testing results was high, but as the epochs increased, the difference between training and testing reached its maximum low. We obtained good segmentation results compared to other state-of-the-art models in our study.

Figures 10(a)–10(h) show training and testing performance curves for accuracy, validation loss, intersection over union, dice coefficient, dice loss, recall, precision, and *F*1 score, respectively. In early epochs, *F*1 score, precision. accuracy, recall, and IoU performance are low, but performance gradually improved without overfitting. In Figure 10(b), it can be seen that validation loss was high in the first five epochs, but after five epochs, it remained below 0 until reaching 100 epochs. In Figure 10(e), it can also be seen that dice loss was high over the first 10 epochs, but after 10 epochs, the difference between training and testing dice loss was minimized.

## 5. Discussion

The proposed model is a supplemented version of the Unet model and includes additional convolution layers at each step of the encoder and decoder and a more weighted connected module. These additions to the conventional Unet model improved its overall efficiency, and the corresponding improvement in results can be seen in Table 1. With the addition of convolution layers and a more weighted module, the proposed model obtained a 1.51%, 4.73%, 2.17%, 1.68%, 1.36%, 1.5% gain as compared to the conventional Unet in terms of accuracy, intersection over union, dice coefficient, recall, precision, and F1score, respectively. Overall, it achieved up to the mark segmentation results in obtaining a dice coefficient score of 92.46%, recall score of 93.01%, F1 score of 93.34%, precision of 93.67%, and Jaccard index of 86.96%. The slightly more weighted connected module obtained sufficient contextual information to ensure better segmentation. Figure 8 shows some instances of the findings acquired that were used to evaluate the performance of the proposed approach for ROI area segmentation. We can see from the data that the suggested model identified the infection well with certain mistakes that are considered insignificant. Furthermore, as shown in Figure 7, the segmentation results obtained from the proposed model are close to the actual ground truth. State-of-the-art comparison in terms of IoU, dice, recall, *F*1 score, precision, and accuracy is presented in Table 3.

The proposed approach used to segment the infection constituted a successful improvement because of the additions we included for intense learning in the baseline approach Unet. The accuracy and robustness of the technique provided were further demonstrated by the evaluation metric results obtained by the model, given in Table 1. Based on these results, we may conclude that the proposed technique outperforms the baseline Unet approach and other state-of-the-art methods. Nevertheless, the model has a large number of parameters which causes an increase in computational cost. In future work, this can be improved further using different techniques involving data augmentation or tuning the hyperparameters.

## 6. Conclusion

This paper proposed a modified model based on Unet architecture to accurately segment COVID-19 lung infections in CT scans. The proposed model, referred to as convUnet, added supplementary convolution layers in encoder and decoder pipelines and improved the convolution module to establish a connection between encoder and decoder pipelines, giving it a major capacity to extract features from the last layer of the encoder pathway and segmentation. The addition of more sets of weights to Unet led to an improvement in its performance. The results obtained from our proposed model proved the efficiency of the convUnet model in segmenting indistinguishable and interconnected areas, as well as the fact that performance evaluation metrics achieved better quantitative results than the basic Unet approach, obtaining a gain in accuracy, intersection over union, dice coefficient, recall, precision and *F*1score of 1.51%, 4.73%, 2.17%, 1.68%, 1.36%, 1.5% respectively. As such, our proposed convUnet method can prove to be beneficial in rapid COVID-19 diagnosis, testing, and quantification of infected areas and provides an overall improvement in COVID-19 lung infection diagnosis.

## Figures and Tables

**Figure 1:** The number of each mask class segmentation in the dataset.

**Figure 2:** Sample dataset images.

**Figure 3:** Architecture of proposed network.

**Figure 4:** Encoder flow diagram.

**Figure 5:** Encoder–decoder and concatenated skip connection flow.

**Figure 6:** Encoder-decoder connected layer block.

**Figure 7:** Actual ground truth of ground glass opacity and predicted ground glass opacity segmentation.

**Figure 8:** Our segmentation model performance.

**Figure 9:** Box plot results.

**Figure 10:** ((a)–(h)) training and testing performance.

**Table 1:** Conventional Unet and improved model convUnet parameters.

Method	Conv-layers	E-D module weight	Batch normalization	Total parameters	Trainable parameters	Optimizer	Learning rate
Unet	16	2	No	31,030,788	31,030,788	Adam	1*e* − 3
convUnet	24	3	Yes	46,773,124	46,755,460	Adam	1*e* − 3

**Table 2:** Best results obtained by proposed model and Unet model over 100 epochs

Method	IoU	Accuracy	Dice-coefficient	*F*1-score	Recall	Precision
Unet	82.83	91.78	90.43	91.82	91.33	92.31
convUnet average value	76.47	83.27	82.52	83.43	82.75	84.11
convUnet	86.96	93.29	92.6	93.34	93.01	93.67
Improvement in convUnet	**4.73↑**	**1.51↑**	**2.17↑**	**1.52↑**	**1.68↑**	**1.36↑**

**Table 3:** State-of-the-art comparison in terms of IoU, dice, recall, *F*1 score, precision, and accuracy.

Source	Models	Acc	IoU	Dice	Recall	*F*1-score	Precision
[26]	3D Unet	—	—	61.0	62.8		74.1
[27]	Encoder-decoder method	—	—	78.6	71.1	78.4	85.6
[28]	AU-Net + FTL	—	—	69.1	81.1	—	—
[29]	Multiple deep CNN	95.23	—	88.0	90.2	—	—
[30]	Imagenet, VGG16 FCN8	—	60.0	75.0	92.0	—	63.0
[31]	DDANet	—	—	77.89	88.40	—	—
[32]	ADID-Unet	97.01	—	80.31	79.73	82.00	84.0
[33]	Semi-Inf-Net	—	—	73.01	72.00	—	—
[12]	Unet	91.78	82.83	90.43	91.33	91.82	92.31
	Ours	93.29	86.96	92.46	93.01	93.34	93.67

## Data Availability

The dataset generated during and/or analysed during the current study are available at http://medicalsegmentation.com/covid19/ and https://doi.org/10.1186/s41747-020-00173-2.
